This article has been retracted.

# The Design of Sports Games under the Internet of Things Fitness by Deep Reinforcement Learning

**DOI:** 10.1155/2022/4623561

**Published:** 2022-05-10

**Authors:** Xiangyu Wang, Chao Liu, Laishuang Sun

**Affiliations:** ^1^School of Social Sport, Shenyang Sport University, Shenyang 110032, Liaoning, China; ^2^Training Department, Chinese Mountaineering Association, Beijing, China

## Abstract

This study explores the application of deep reinforcement learning (DRL) in the Internet of Things (IoT) sports game design. The fundamentals of DRL are deeply understood by investigating the current state of IoT fitness applications and the most popular sports game design architectures. The research object is the ball return decision problem of the popular game of table tennis robot return. Deep deterministic policy gradients are proposed by applying DRL to the ball return decision of a table tennis robot. It mainly uses the probability distribution function to represent the optimal decision solution in the Markov Model decision process to optimize the ball return accuracy and network running time. The results show that in the central area of the table, the accuracy of returning the ball is higher, reaching 67.2654%. Different tolerance radii have different convergence curves. When *r* = 5 cm, the curve converges earlier. After 500,000 iterations, the curve converges, and the accuracy rate is close to 100%. When *r* = 2 cm and the number of iterations is 800,000, the curve begins to converge, and the accuracy rate reaches 96.9587%. When *r* = 1 cm, it starts to converge after 800,000 iterations, and the accuracy is close to 56.6953%. The proposed table tennis robot returns the ball in line with the requirements of the actual environment. It has practical application and reference value for developing IoT fitness and sports.

## 1. Introduction

With the development of information technology and the popularization of IoT fitness, various sports, somatosensory, and virtual reality fitness games that combine artificial intelligence (AI) and sensor technology have been developed and received widespread attention [1]. Many application problems in AI require algorithms as support. In fitness games, game characters can make decisions and perform actions at every moment [2]. Go needs to calculate where on the board to place the pieces to defeat the opponent. Autonomous driving requires algorithms to determine how to perform each action to ensure driving safety. The table tennis robot needs an algorithm to help determine the ball's location to make an accurate return. They all need to make decisions and actions by certain conditions to achieve the expected goals [3–5]. Deep reinforcement learning (DRL) has powerful advantages in this type of intelligent decision-making needs [6].

Table tennis is a sport, and precise movement control is significant. Yang, et al. (2021) [7] proposed a ball hitting strategy to ensure the ideal “target landing position” and “super clear height”. These are two key indicators for evaluating the quality of a shot. To overcome the spin speed challenge, they also developed a spin speed estimation method by DRL in their research [8]. This method can predict the relative spin speed of the ball and accurately knock it back by iteratively learning the interaction between the robot and the environment. Although most motion data-driven models have nonlinear structure and high predictive performance, these models are sometimes intricate to interpret the ball's trajectory. Fujii (2021) [9] used data to drive analysis to quantitatively understand behaviors in team sports such as basketball and football. They introduced two main methods for understanding the behavior of such multiagents: extracting easy-to-interpret features or rules from data and generating and controlling behavior in an intuitive and easy-to-understand manner. Noninvasive systems for data acquisition were created through computer vision, image processing, and software teaching techniques. This system may help identify players' positions and roles in basketball games. Jiang, et al. (2021) [10] proposed a video framework by deep learning to build a player position system. They used traditional regression techniques to determine each person's position so that the player moves toward the ball position. Therefore, the application of DRL in sports can help players accurately control the movement process. The research provides new ideas for the IoT sports game fitness field.

Methods of literature research and algorithm validation are adopted. The application status of Internet of Things (IoT) fitness sports games is deeply studied. The main contribution and innovation lie in using DRL to optimize the performance of sports games and improve the precision and accuracy of the table tennis robot returning the ball. In addition, the proposed intensive deep learning network can improve the ball return accuracy of the table tennis robot. The purpose of DRL is to speed up the convergence of the regression on curve. In the 20 rounds of testing, the average output time of a single ball return action of the network model is shorter. This shows that the model can meet the real-time response requirements of the table tennis robot to the decision to return the ball. The proposed deep deterministic policy gradient is used to optimize the accuracy of the table tennis robot's return decision, which can achieve good model detection results.

## 2. Materials and Methods

### 2.1. DRL

Machine learning uses data or experience to improve algorithm performance indicators. It is divided into supervised learning, semi-supervised learning, unsupervised learning, and reinforcement learning [11]. Reinforcement learning (RL) is a type of machine learning. It belongs to unsupervised learning and can imitate the basic way of human learning [12]. Its composition includes agent, reward, environment, state, and action [13]. The relationship between the various components of RL is shown in Figure 1. RL collects corresponding state, action, and reward samples for trial-and-error learning through the interaction between the agent and the environment. Then, it continuously improves its strategy to obtain the most considerable cumulative reward. Finally, the optimal solution of its action strategy is accepted, so that the accumulated bonus reaches the maximum. So, it is widely used in intelligent learning [14–16].

DRL is an enhanced version of RL, a product of deep learning and RL. It not only integrates deep learning's strong understanding of perception problems such as vision but also has the decision-making ability of RL and realizes end-to-end learning [17]. It uses artificial neural networks to replace the action-value function in RL [18]. The neural network has a robust, expressive ability and can autonomously search for features. Agents can accurately predict and judge in complex environments. It links deep learning and RL, uses agents to make decisions, and uses deep learning methods to extract features from state vectors. Agents are expressed in images, and deep learning methods operate on them. The agent uses RL to make decisions and allocate resources. The emergence of DRL makes RL technology move from theory to practice and solves complex problems in real-life scenarios. For example, in games, DRL can obtain a large amount of sample data at almost no cost through continuous trial and error and improve the final training effect.

### 2.2. IoT Smart Sports Game Design

Smart sports are applying modern information technologies such as IoT, cloud computing, and AI in sports and fitness. It is often used in sports wearable equipment, fitness equipment, fitness venues, and national fitness competitions [19]. In Figure 2, compared to traditional fitness clubs, smart fitness uses IoT intelligent conventional fitness equipment, Internet data, and mobile terminals to achieve online and offline integration [20–22]. Users can use their mobile phones to scan the QR code or swipe the card to open the equipment for exercise. The device will automatically record the user's height, weight, exercise duration, number of exercises, etc., and upload the exercise data to the app. The app will give an exercise evaluation report and suggestions for improving fitness actions. Compare and analyze historical exercise data, and the app will provide recommendations for the next exercise plan by the user's exercise goals. The designed fitness venue has high operating efficiency, a small footprint, low investment, and unlimited business hours. This kind of fitness center management is more lightweight and clearer. It has low labor costs and low management difficulty and can provide users with personalized and differentiated fitness services.

Interactive and immersive experience sports games increase users' interest and motivation for fitness—the combination of virtual reality and sports upgrades the hardware of ordinary sports games. The hardware is intelligent to record life and sports data more accurately. The innovative equipment can reduce the probability of sports injuries and improve sports performance by upgrading materials. Artificial Intelligence (AI) is standard for most games. Any game with nonplayer character (NPC) [23] needs the support of the AI system. AI makes NPCs come to life, and players have an immersive feeling in the game world. Virtual reality (VR) fitness games can assist fitness and make fitness fun. The components of the VR game are shown in Figure 3:

In Figure 3, in virtual reality games, users can feel the feeling of fighting and constant movement. Different exercise programs arranged by professional fitness trainers will track the calories burned by the user over the exercise time. Such virtual reality fitness games are usually bright graphics and exciting music. All designs can help users concentrate on achieving the best fitness effect. Different levels of fitness users have various courses designed. Users can also upload their music to get a tailor-made exercise program. Dance fitness games are very energetic. It can encourage players to use all their muscles. Rhythm plays an essential role in the fun. Each level is a dance designed by professional dancers. The posture ranges from single-arm to cross-arm to tapping, lunge, squatting, and other dance moves, allowing users to experience stage dancing in an immersive manner.

### 2.3. Decision Analysis of Return Ball of Table Tennis Robot by DRL

In table tennis sports, ball return decision-making refers to the question of what posture and speed should be used to hit the ball in the case of determining the motion state of the incoming ball and the expected impact position. In previous studies, nonlinear optimization methods were often used to solve the robot end pose. This method is only suitable for nonrotating ball return decisions. It needs to be further studied for the handling of complex situations. DRL has advantages in decision-making and planning. RL uses Markov decision process (MDP) [24] as a mathematical model, expressed as (*S*, *A*, *T*, *R*, *γ*). Among them, *S* represents the state collection, *A* represents a collection of actions, *T* indicates the probability of performing a movement in the current state to transition to a certain state, *R* indicates the corresponding reward, *γ* ∈ [0,1] represents the discount coefficient, which indicates the importance of future and current earnings. The purpose of MDP is to find the optimal solution of a strategy *π* to ensure that in the state of *s*, the profit obtained *R*[*T*] by the selected action *a* reaches the maximum, as shown in:

(1) $$\begin{array}{c} R\left[T\right]=\sum_{t=0}^{T}r^{t}R_{a_{i}}\left(s_{t},s_{t+1}\right). \end{array}$$

When *r*=0, only immediate benefits are considered. When *r*=1, immediate benefits and long-term benefits are of equal importance.

DRL has advantages as unsupervised learning. RL can generate data autonomously during the training process and does not require complex labeling work with the help of the income function. Deep deterministic policy gradient (DDPG) is a DRL algorithm. It mainly represents the optimal decision-making solution in MDP decision-making through the probability distribution function. The process of generating actions is random. The specific algorithm implementation framework is shown in Figure 4:

DDPG is used to deal with the decision-making problem of the ball return of the table tennis robot. The specific implementation framework is designed, and the structure diagram is shown in Figure 5. The service machine in the frame randomly sends out different states of ping-pong balls. After the table tennis is launched, the trajectory model of rotating table tennis and the collision model of table tennis will get the state of the ball in the preset hitting plane through the operation *s*. Meanwhile, this state is output to the decision-making algorithm of the table tennis robot. When the algorithm receives the table tennis status *s*, it gives the action *a* that should be executed according to the current state of the ball. It transmits the execution parameter data information to the table tennis simulation environment. Table tennis simulates a racket in a simulated environment will be calculated according to the state of the table tennis robot *s* and the motion of table tennis *a* after they were back. Then, it calculates the actual drop point of the ping-pong ball being hit by the trajectory model of the rotating ping-pong ball. Finally, the immediate benefits of this set of experiments are obtained after comparing with the expected landing point. This set of ball return experiments is completed.

Two sets of coordinate systems of table tennis table and racket are set in the simulation environment of table tennis. The table tennis table coordinate system serves the trajectory model of the rotating table tennis and the collision model of the table. The racket coordinate system is used for calculations related to the collision model of the table tennis racket. Three models are used in the simulation environment. The collision model of the rotating ping-pong ball and the table adopts the collision model of the rotating ping-pong ball by optical measurement. Under normal circumstances, the entire collision process is simplified to a momentary state change, or the friction coefficient is simplified to a linear quantity or even a constant. The dynamic collision process between the rotating ping-pong ball and the table is used for mechanism analysis. The collision process between the rotating ping-pong ball and the table is a series of continuous physical transfer processes. Its duration has nothing to do with the state of motion of the incoming ball. The mean value theorem [25] and the law of momentum conservation are combined to obtain the expression of the collision model as Eqs. (2) - (7):

(2) $$\begin{array}{c} \overset{+}{\underset{z}{v}}=-\alpha_{z}\overset{-}{\underset{z}{v}}, \end{array}$$

(3) $$\begin{array}{c} \overset{+}{\underset{x}{v}}=\overset{-}{\underset{x}{v}}+f_{\mu x}\left({\overset{⟶}{v}}_{-},{\overset{⟶}{w}}_{-}\right)\left(\overset{+}{\underset{z}{v}}\overset{-}{\underset{z}{-v}}\right), \end{array}$$

(4) $$\begin{array}{c} \overset{+}{\underset{y}{v}}=\overset{-}{\underset{y}{v}}+f_{\mu y}\left({\overset{⟶}{v}}_{-},{\overset{⟶}{w}}_{-}\right)\left(\overset{+}{\underset{z}{v}}\overset{-}{\underset{z}{-v}}\right), \end{array}$$

(5) $$\begin{array}{c} \overset{+}{\underset{x}{w}}=\overset{-}{\underset{x}{w}}+m{f_{D_{x}}f}_{\mu x}\left({\overset{⟶}{v}}_{-},{\overset{⟶}{w}}_{-}\right)\left(\overset{+}{\underset{z}{v}}\overset{-}{\underset{z}{-v}}\right), \end{array}$$

(6) $$\begin{array}{c} \overset{+}{\underset{x}{w}}=\overset{-}{\underset{y}{w}}+m{f_{D_{x}}f}_{\mu y}\left({\overset{⟶}{v}}_{-},{\overset{⟶}{w}}_{-}\right)\left(\overset{+}{\underset{z}{v}}\overset{-}{\underset{z}{-v}}\right), \end{array}$$

(7) $$\begin{array}{c} \overset{+}{\underset{z}{w}}=\overset{-}{\underset{z}{w}}+f_{M_{N}}. \end{array}$$

Among them, *v*_*x*_^+^, *v*_*y*_^+^, *v*_*z*_^+^, respectively, represent the respective movement speeds of the rotating ping-pong ball in the three coordinate axis directions *x*, *y*, *z* after the collision, *v*_*x*_^−^, *v*_*y*_^−^, *v*_*z*_^−^, respectively, represent the respective movement speeds of the rotating ping-pong ball in the respective *x*, *y*, *z* directions before the collision, *w*_*x*_^+^, *w*_*y*_^+^, *w*_*z*_^+^, respectively, represent the respective rotation speeds of the rotating ping-pong ball in the *x*, *y*, *z* directions after the collision, *w*_*x*_^−^, *w*_*y*_^−^, *w*_*z*_^−^, respectively, represent the rotation speed of the rotating ping-pong ball in each *x*, *y*, *z* direction before the collision, *α*_*z*_, *f*_*μx*_,*f*_*μy*_, *f*_*M*_*N*__,*f*_*D*_*x*__ represent the collision coefficient related to the rotation speed and flight speed of the incoming ball, and *m* represents the quality of the ping-pong ball in the experiment.

The derivation process of the collision model between the rotating ping-pong ball and the racket is almost the same as the derivation process of the table collision model except for the different coordinate systems. The table coordinate system is converted to the rotation matrix of the racket coordinate system for derivation. The expression of the collision model is shown in Eqs. (8) - (13):

(8) $$\begin{array}{c} \overset{+}{\underset{z}{v}}=-\alpha_{z}\overset{-}{\underset{z}{v}}+\beta_{z}\overset{\text{racket}}{\underset{z}{v}}, \end{array}$$

(9) $$\begin{array}{c} \overset{+}{\underset{x}{v}}=\overset{-}{\underset{x}{v}}+f_{\mu x}\left({\overset{⟶}{v}}_{-},{\overset{⟶}{w}}_{-},{\overset{⟶}{\text{v}}}_{\text{racket}}\right)\left(\overset{+}{\underset{z}{v}}\overset{-}{\underset{z}{-v}}\right), \end{array}$$

(10) $$\begin{array}{c} \overset{+}{\underset{y}{v}}=\overset{-}{\underset{y}{v}}+f_{\mu y}\left({\overset{⟶}{v}}_{-},{\overset{⟶}{w}}_{-},{\overset{⟶}{v}}_{\text{racket}}\right)\left(\overset{+}{\underset{z}{v}}\overset{-}{\underset{z}{-v}}\right), \end{array}$$

(11) $$\begin{array}{c} \overset{+}{\underset{x}{w}}=\overset{-}{\underset{x}{w}}+\frac{m}{I}f_{\mu \text{ lx}}\left({\overset{⟶}{v}}_{-},{\overset{⟶}{w}}_{-},{\overset{⟶}{v}}_{\text{racket}}\right)\left(\overset{+}{\underset{z}{v}}\overset{-}{\underset{z}{-v}}\right), \end{array}$$

(12) $$\begin{array}{c} \overset{+}{\underset{x}{w}}=\overset{-}{\underset{y}{w}}+\frac{m}{I}f_{\mu \text{ ly}}\left({\overset{⟶}{v}}_{-},{\overset{⟶}{w}}_{-},{\overset{⟶}{v}}_{\text{racket}}\right)\left(\overset{+}{\underset{z}{v}}\overset{-}{\underset{z}{-v}}\right), \end{array}$$

(13) $$\begin{array}{c} \overset{+}{\underset{z}{w}}=\overset{-}{\underset{z}{e_{z}w}}, \end{array}$$

*v*_racket_ represents the speed of the racket, *f*_*μx*_,*f*_*μy*_, *f*_*μ* lx_,*f*_*μ* ly_, *α*_*z*_,*β*_*z*_, *e*_*z*_ represent the collision coefficient related to the speed of the racket, the flight speed of the rotating ping-pong ball, and the rotation speed of the ping-pong ball. *I* represents the moment of inertia of the rotating ping-pong ball. Due to the uneven mass distribution of the ping-pong ball during the collision, the moment of inertia of the rotating ping-pong ball also expresses the variables related to the above three motion states. The extended continuous motion model uses the trajectory model of the rotating table tennis ball to estimate the optimal state of the rotating ball and the trajectory prediction model. Through the force analysis of gravity, air resistance, and other comprehensive forces in the process of table tennis. The Fourier series fitting the attenuation curve of the relationship between speed and time during the movement of rotating table tennis is used to derive the trajectory model of table tennis.

The hitting plane is designed in advance to plan the path of the rotating table tennis ball. The intersection of the trajectory of the table tennis ball and the hitting plane is the hitting point. In the simulated environment, the “ball machine” will continue to generate random incoming balls. The three models in the background are used to calculate the motion state of the rotating ping-pong ball on the predesigned hitting plane, which is transmitted to the decision-making algorithm. Therefore, the input of the DDPG algorithm is the motion state *s* of the rotating table tennis ball on the present hitting plane, as shown in:

(14) $$\begin{array}{c} s={\left[{\overset{⟶}{p}}_{\text{input}},{\overset{⟶}{v}}_{\text{input}},{\overset{⟶}{w}}_{\text{input}},{\overset{⟶}{p}}_{\text{target}}\right]}^{T}. \end{array}$$

In (14): the various equations represent:

(15) $$\begin{array}{c} {\overset{⟶}{p}}_{\text{input}}={\left[\begin{array}{ccc} p_{x} & p_{y} & p_{z} \end{array}\right]}^{T},\\ {\overset{⟶}{v}}_{\text{input}}={\left[\begin{array}{ccc} v_{x} & v_{y} & v_{z} \end{array}\right]}^{T},\\ {\overset{⟶}{w}}_{\text{input}}={\left[\begin{array}{ccc} w_{x} & w_{y} & w_{z} \end{array}\right]}^{T},\\ {\overset{⟶}{p}}_{\text{target}}={\left[\begin{array}{cc} p_{\text{tx}} & p_{\text{ty}} \end{array}\right]}^{T}, \end{array}$$

${\overset{⟶}{p}}_{\text{input}}$ represents the spatial position of the table tennis ball in the table coordinate system, ${\overset{⟶}{v}}_{\text{input}}$ represents the flying speed of the table tennis ball, ${\overset{⟶}{w}}_{\text{input}}$ represents the rotation speed of the table tennis ball, and ${\overset{⟶}{p}}_{\text{target}}$ represents the expected landing position of the table tennis ball. The goal of table tennis decision planning is the end motion state of the table tennis robot, which is the final output of the network model. On the premise that other factors have been determined, the position, posture and speed of the racket are determined. So, the output action is expressed as

(16) $$\begin{array}{c} \overset{⟶}{a}={\left[\begin{array}{c} {\overset{⟶}{n}}_{r} \end{array}\right]}^{T}. \end{array}$$

(17) $$\begin{array}{c} {\overset{⟶}{v}}_{r}={\left[\begin{array}{cc} v_{\text{ry}} & v_{\text{rz}} \end{array}\right]}^{T}, \end{array}$$

${\overset{⟶}{v}}_{r}$ represents the speed of the racket in the axis direction *x*, *y*, *z* of the table coordinate system, and ${\overset{⟶}{n}}_{r}$ represents the vector used to represent the position and posture of the table tennis racket at the hitting point in the table coordinate system. Since the impact of the front and back of the table tennis racket on the hitting result can be ignored, *n*_*y*_ in ${\overset{⟶}{n}}_{r}$ is set to -1.

When the DRL-based DDPG algorithm is used for network training, the return function needs to consider the accuracy and safety of the ball return, as shown in

(18) $$\begin{array}{c} R=-k\left(\left\|p-p_{\text{target}}\right\|+\left\|z_{\text{act}}-z_{\text{net}}\right\|\right). \end{array}$$

In (18), *k* represents the weight coefficient, *p* represents the actual return point of the ping-pong ball, *p*_target_ represents the expected fall point of the incoming ball, *z*_act_ represents the height of the ball from the table when it passes the net during the current return process, and *z*_net_=0.27*m* represents the height of the ping-pong net. The ball return decision problem is a single-step MDP decision problem, so the median function network and strategy network optimization of the DDPG algorithm only need to use the estimation network.

The proposed DDPG algorithm is simulated. The operating hardware environment used is a 24-core Inter X5670 computer. It is developed by the open-source framework TensorFlow and the optimizer uses AdamOptimizer. The step length of each iteration update is within a range, so there will be no varying learning step length. In the simulated environment, the athletic ability and state of table tennis are limited. The state of random incoming balls generated by the ball machine in the simulated environment is restricted. The state of unexpected balls is kept within a reasonable range. Meanwhile, the action output must also be constrained. The content of motion status is set as shown in Table 1:

Accuracy is used as a measure to evaluate the accuracy of the DDPG network model. It means that in a set of ball return tests, the return ball falls within a circular plane with the expected fall point as the center and *r* as the radius. *r* indicates the error value of the allowable range. In the actual test, the capacity of the scheduled drop point is further divided according to the *x*-axis and *y*-axis directions, and a test point is selected at an interval of 1 cm. The plane of the entire return ball landing point is divided into 160 × 80 small areas. Among them, it contains 160 × 81 tests point. Perform 5000 ball return tests for each test point and record the actual drop point position of each return ball. The accuracy of the ball return for each expected landing is calculated. The maximum number of iterations is set to times. Different iteration times are selected for performance analysis.

The real-time test process of the DDPG network model is shown in Figure 6:

During the test, set the number of test rounds *M*=20, the test times of the model *N*=20 in each round, and the time consumed in each round of network model testing.

## 3. Results and Discussion

### 3.1. Comparison of Ball Return Accuracy of DDPG Network Model under Different Iterations

According to the center region of the table, the middle region, and the edge region of the table, the drop point area of the return ball is divided into three areas: area 1, area 2, and area 3. The error value of the allowed range is set as *r* = 1 cm. The return accuracy results of different regions are shown in Figure 7:

In Figure 7, in most cases, area 1, namely the center area of the table, has a high return accuracy rate of 67.2654%. Area 3, namely the edge area of the table, has a low accuracy rate of 0.9756%. With the number of iterations, the overall return accuracy showed a rising trend.

The convergence curve results of the network model as the number of iterations increases are shown in Figure 8:

In Figure 8, convergence curves of different allowable error radii are different. When *r* = 5 cm, it converges earlier and begins to converge when the number of iterations is 500,000, with an accuracy of nearly 100%. When *r* = 2 cm, it starts to converge when the number of iterations is 800,000, and the accuracy rate reaches 96.9587%. When *r* = 1 cm, it begins to converge when the number of iterations is 800,000, and the accuracy is close to 56.6953%. In a formal table tennis game, the diameter of a table tennis ball is 4 cm. It shows that the depth deterministic strategy gradient algorithm DDPG model return accuracy rate can reach the error within a table tennis diameter. Therefore, the model can meet the requirements of the table tennis robot training system for the accuracy of the ball return.

DDPG real-time test results of the network model.

The time consumption results of the DDPG network model are shown in Figures 9 and 10:

In Figure 9, in the longest round of testing, the average network time is 0.49279 ms. In the shortest round of testing, the average network time is 0.4004 ms. In the 20 rounds of testing, the average output time of a single ball return action of the network model is 0.4658 ms. In addition, in Figure 10, in the most extended round of testing, the time-consuming statistical average of the test network is the shortest test, 0.1 ms. This shows that the model can meet the real-time response requirements of the table tennis robot to the decision to return the ball.

## 4. Conclusions

With the popularity of IoT fitness, various sports are moving towards digital and intelligent development. This study combines the current status of IoT innovative sports projects, analyzes the reasons for the popularity of sports games based on advanced information technology, and proposes a fitness model for sports-oriented immersive games. After the principles of DRL and its advantages in intelligent learning are understood, DRL is applied to the training of table tennis robots in sports competitions. The deep deterministic policy gradient algorithm network model of DRL can effectively improve the accuracy of the table tennis robot's return decision and can meet the real-time requirements of the table tennis robot's return decision. Some scholars have conducted research based on the significance of DRL and neuroscience. Deep learning is used as the basis for modeling brain function. The results show that deep RL provides an agent-based framework for studying how rewards shape representations and how representations, in turn, shape learning and decision-making. This is consistent with the results obtained, showing that deep learning can improve the accuracy of IoT fitness sports games. However, there are still some deficiencies to be improved. The proposed algorithm is only run in a simulated environment, and the ball return practice in the natural environment is also required to verify the accuracy. In addition, due to the delay and error of system execution, the actual execution process may affect the final ball return accuracy. In future research, the virtual environment will need to be further trained, and the appropriate algorithm optimization range will need to be selected to improve the accuracy of the algorithm further.

## Figures and Tables

**Figure 1:** The relationship between the environment of RL and the agent.

**Figure 2:** Smart fitness club operating model.

**Figure 3:** Virtual reality game module composition.

**Figure 4:** DDPG algorithm framework diagram.

**Figure 5:** Table tennis robot returns the ball decision frame diagram.

**Figure 6:** DDPG real-time testing process of the network model.

**Figure 7:** Return accuracy results in different areas.

**Figure 8:** Convergence curve of ball accuracy under different allowable errors.

**Figure 9:** Network time-consuming statistics for 1∼10 tests.

**Figure 10:** Network time statistics when the number of tests is 11 to 20.

**Table 1:** Constraint table of the incoming ball state of the present hitting plane.

Experimental variables	Ranges
Px	[-50 cm, +50 cm]
Py	121.3 cm
Pz	[0, 50 cm]
Vx	[-50 cm/s, +50 cm/s]
Vy	[250 cm/s, 650 cm/s]
Vz	[-50 cm/s, +50 cm/s]
Wx	[-100 rad/s, +100 rad/s]
Wy	10 rad/s
Wz	[-100 rad/s, +100 rad/s]
Ptx	[-80 cm, +80 cm]
Pty	[-110 cm, -30 cm]
Nx	[-0.5, 0.5]
Ny	-1
Nz	[-0.5, 0.5]

The range of motion variables generated by the simulated environment is -50 cm/*s* < vrx<50 cm/s, -300 cm/*s* < vry<0 cm/s, -50 cm/*s* < vrx<50 cm/s.

## Data Availability

The data used to support the findings of this study are available from the corresponding author upon request.
